The article "Lipidomics, transcription analysis, and hormone profiling unveil the role of CsLOX6 in MeJA biosynthesis during black tea processing" was retracted in 2024. Reasons: no approval from a third party; concerns about the data; concerns about the authorship.

# Lipidomics, transcription analysis, and hormone profiling unveil the role of *CsLOX6* in MeJA biosynthesis during black tea processing

**DOI:** 10.1093/hr/uhae032

**Published:** 2024-01-30

**Authors:** Gaoyang Zhang, Jingjing Wei, Linyan Li, Dandan Cui

**Affiliations:** School of Biological Engineering, Henan University of Technology, Zhengzhou 450001, China; School of Biological Engineering, Henan University of Technology, Zhengzhou 450001, China; College of Advanced Interdisciplinary Science and Technology, Henan University of Technology, Zhengzhou 450001, China; State Key Laboratory of Tea Plant Biology and Utilization, College of Tea and Food Science and Technology, Anhui Agricultural University, Hefei, 230036, China

## Abstract

Jasmonates, such as jasmonic acid (JA) and methyl jasmonate (MeJA), are crucial aspect of black tea quality. However, lipids species, hormones, and genes regulated mechanism in the jasmonate biosynthesis during black tea processing are lacking. In this study, we employed lipidomics, hormone metabolism analysis, and transcriptome profiling of genes associated with the MeJA biosynthesis pathway to investigate these factors. The contents of lipids GLs, PLs, and TAG are decreased, accompanied by the main lipids species reduced during black tea processing. Galactolipids, primarily 34:3/36:6/36:3 DGDG and 36:6/36:5/36:4 MGDG, are transformed into massive MeJA and JA in black tea processing, accompanied by the decreased SA, MeSA, IAA, and BA and increased zeatin. Additionally, the transcriptional activity of the primary genes in MeJA biosynthesis pathway exhibited downregulated trends except for *AOS* and *OPR* and non-primary genes tend to be a little high or have fluctuation of expression. Coordinated expression of main *CsHPL (TEA008699), CsAOS (TEA001041)*, and Cs*JMT (TEA015791)* control the flow of lipids degradation and MeJA production. A strong infected reduction of a key lipoxygenase gene, *CsLOX6 (TEA009423)*, in tea buds significantly reduced the level of jasmonates and expression of downstream genes, accompanied by SA, MeSA level rising, and ABA declining. We have identified a key *CsLOX6*, as well as established galactolipids, mainly 34:3/36:6/36:3 DGDG and 36:6/36:5/36:4 MGDG, sources for MeJA biosynthesis regulated by dynamics hormone and controlled by coordinated expressed *CsHPL (TEA008699), CsAOS (TEA001041)*, and *CsJMT (TEA015791)*. Our findings provide a theoretical basis for breeding high-quality black tea and offer valuable insights for improving processing methods.

## Introduction

Black tea encompasses one of the most traditional non-alcoholic beverages consumed worldwide due to its health benefit, taste, and aroma [1, 2]. Black tea is made through the full fermentation of the leaves of *Camellia sinensis* (Theaceae), which involves four distinct stages: withering, rolling, fermentation, and drying [3, 4]. Jasmonate species, including 12-oxo-phytodienoic acid (OPDA), dinor-phytodienoic acid (dnOPDA), jasmonic acid (JA), and methyl jasmonate (MeJA), have been related to different developmental processes and stress responses in plants [5, 6]. MeJA is a well-characterized fatty acid-derived cyclopentanone aroma compound and cellular signal that triggers and modulates the synthesis of specialized metabolites in a wide range of plant groups [7]. Because aroma is a major aspect of tea quality, MeJA has been widely applied in promoting food quality, especially to change the aroma qualities of flavor profiles during the processing of green, oolong, and black teas [2, 8, 9]. Black tea manufacturing encompasses a complex biological process that causes widespread damage to membrane structures as the tea shoots are dehydrated and broken down mechanically as well as by the action of enzymes during processing [10, 11]. Therefore, the role of hormones related to plant defense during tea processing warrants an analysis. The role of MeJA during black tea processing may affect its beverage quality and health properties.

The article "Lipidomics, transcription analysis, and hormone profiling unveil the role of CsLOX6 in MeJA biosynthesis during black tea processing" was retracted in 2024. Reasons: no approval from a third party; concerns about the data; concerns about the authorship.

Tea lipids profiling in preharvest and postharvest leaves have been studied in previous research [12]. The lipids types encompass fatty acids, glycerols, phospholipids, glycolipids in tea leaves, which are similar to major plant lipids, such as *Arabidopsis* [9, 12]. The proportion of total lipid content in fresh tea leaves is about 4–9% of dry weight [13]. The membrane glycoglycerolipids include monogalactosyldiacylglycerol (MGDG), digalactosyl diacylglycerol (DGDG), sulfoquinovosyldiacylglycerol (SQDG), and glycerophospholipids contain phosphatidylcholine (PC), phosphatidylethanolamine (PE), phosphatidylglycerol (PG), phosphatidylinositol (PI), phosphatidylserine (PS), and phosphatidic acid (PA).The stored acylglycerolipids are composed of triacylglycerol (TAG) and diacylglycerol (DAG). PC, PE, MGDG, SQDG, and TAG are major lipid types in tea leaves [12, 14]. Abotic factors, such as shading treatment, low temperature, nitrogen fertilizer treatment, abscisic acid, methyl jasmonate spraying, and biotic factors such as herbivores attack, tea tortrix, *Ectropis obliqua* suck, *Colletotrichum camelliae* infection affect lipids composition in preharvest tea leaves [9, 12, 13, 15].

It has been established that the fatty acid substrate for JA biosynthesis is α-linolenic acid (18:3) released from the sn_1_ position of galactolipids of chloroplast membranes by phospholipase 1 (PLA1) hydrolysis, which is activated by certain stimuli [5, 6, 16]. The α-linolenic acid is oxygenated by lipoxygenase (LOX) to form a peroxidation product (9Z,11E,13S,15Z)-13-hydroperoxy-9,11,15-octadecatrienoic acid (13-HPOT) via the octadecanoid pathway [6, 17]. The hydroperoxide 13-HPOT is cyclized to OPDA by the sequential action of allene oxide synthase (AOS) and allene oxide cyclase (AOC) in the plastids [18]. Following, JA is synthesized from OPDA through reduction of a double bond and three rounds of β-oxidation by OPDA reductase (OPR) and acyl-CoA-oxidase (ACX) in the peroxisome [5, 16]. JA is then further catabolized to form its volatile counterpart, MeJA by the JA carboxyl methyltransferase (JMT) [17]. Additionally, a cytoplasmic pathway for JA biosynthesis has also been described [18]. OPDA and dnOPDA can occur as free acids in *Arabidopsis* and also as esters of complex lipids, the so-called arabidopsides, which include derivatives of MGDG and DGDG, respectively, which contain one or two chains of OPDA and/or dnOPDA [19, 20]. Thus, the alternative pathway for JA biosynthesis is expected to sequentially involve LOX, AOS, AOC, and PLA enzymatic functions in the plastids [20].

The article "Lipidomics, transcription analysis, and hormone profiling unveil the role of CsLOX6 in MeJA biosynthesis during black tea processing" was retracted in 2024. Reasons: no approval from a third party; concerns about the data; concerns about the authorship.

Although knowledge of lipid degradation into MeJA has been known for a long time, little research has been carried out to demonstrate the connection between MeJA biosynthesis and lipid profile during black tea processing [10]. By the same token, the gene expression profile of the MeJA biosynthesis pathway during black tea processing has not been properly addressed yet. The present investigation reports the composition of neutral lipids, glycolipids, lysophospholipids, and phospholipids, along with their fatty acid forms, at different stages of black tea manufacture. By analysing the transcriptional changes of MeJA biosynthesis-related genes and profiling jasmonates during black tea processing, we identify and confirm that *CsLOX6* is clearly associated with MeJA formation. This information is not only helpful but also critical to breed tea varieties aiming for high-quality beverages.

**Figure 1:** Glycerolipid profiling during black tea processing. **(a)** Appearance of leaves during black tea processing. **(b)** TLC separation of lipids from leaves during black tea processing. **(c)** Total glycerolipids levels in leaves during black tea processing. **(d)** Glycerolipids percentage of total signal in fresh leaves. **(e)** Lysophospholipid profiles during black tea processing. **(f)** Principal component analysis (PCA) with glycerolipidic data during black tea processing. Score plot: R^2^ X = 0.622, Q^2^ = 0.469. **(g)** The profiles of glycerolipids species in leaves during black tea processing. The heat maps of Z score-normalized values were shown. DGDG: digalactosyl diacylglycerol; LPC: lysophosphatidylcholine; LPE: lysophosphatidylethanolamine; LPG: lysophosphatidylglycerol; MGDG: monogalactosyl diacylglycerol; PA: phosphatidic acid; PC: phosphatidylcholine; PE: phosphatidylethanolamine; PG: phosphatidylglycerol; PI: phosphatidylinositol; PS: phosphatidylserine; SQDG: sulfoquinovosyldiacylglycerol. The values are presented as means ± S.D (*n* = 4 or 5). All ^*^ and ^**^ denote significance at *P* < 0.05 and *P* < 0.01, respectively, compared with fresh samples based on Student’s *t-*test.

The article "Lipidomics, transcription analysis, and hormone profiling unveil the role of CsLOX6 in MeJA biosynthesis during black tea processing" was retracted in 2024. Reasons: no approval from a third party; concerns about the data; concerns about the authorship.

## Results

### Glycerolipid profiling in leaves during black tea processing

To further understand the profiles in the structural membrane lipids during black tea processing, a lipidomic analysis was carried with electrospray ionisation-liquid chromatography tandem mass spectroscopy (LC-ESI-MS/MS) to profile polar membrane glycerolipids, including galactolipids (GLs) and phospholipids (PLs). The results showed that DGDG, MGDG, SQDG, PG, PC, PE, PI, PS, PA were present in leaves over different black tea stages (Fig. 1; Fig. S1–3, see online supplementary material). Although glycerolipids species did not change qualitatively during black tea processing, i.e., no new forms appeared during processing, their contents varied broadly (Fig. 1c). Mostly, the total contents of the GLs, DGDG, MGDG, and SQDG dropped almost linearly during processing, with dried samples containing 93%, 93%, and 80% reduction of the starting amounts, respectively (Fig. 1c). Regarding the PL species, the contents of PG, PC, PE, and PI decreased steadily during processing, except for a small increase during the rolling step, and dried samples contained 75%, 89%, 82%, 80% less than the original samples, respectively, for each PL form (Fig. 1c). The PS trend was similar to GL during processing, declining about 94% in dried samples compared to fresh samples (Fig. 1c). PA content fluctuated during processing, and dried samples showed an 86% decrease of that in fresh samples (Fig. 1c).

The decrease in content observed for the main DGDG, MGDG, and SQDG species during processing compared to their total content with the 34:3, 36:6 forms having decreased 95% for both DGDG species in the dried samples compared to fresh samples (Fig. 1g; Fig. S2a–c, see online supplementary material). The secondary DGDG forms, 34:2, 34:1, 36:5, 36:4, and 36:3, decreased by 91%, 89%, 90%, 91%, and 93%, respectively, in dried samples compared to the fresh ones (Fig. 1g; Fig. S2a, see online supplementary material). Although the amounts of the remaining DGDG species were small, the proportion also sharply dropped in drying samples. For examples, 38:6 DGDG decreased by 95% in drying samples (Fig. 1g; Fig. S2a, see online supplementary material). The highest content of all glycerolipids species, 36:6 MGDG, declined sustainably during processing, with dried samples showing a 94% reduction of the values of fresh samples (Fig. 1g; Fig. S2b, see online supplementary material). All other MGDG species also decreased sharply, such as 36:5 and 36:4 MGDG, which showed respective decreases of 92% and 91% in dried samples compared to freshly harvested material (Fig. 1g; Fig. S2b, see online supplementary material). For SQDGs, contents of the main 34:3, 34:2, and 34:1 SQDG species decreased respectively by 86%, 81%, and 73% in dried samples along with the other SQDG species, 36:5, 36:4, and 36:3, which also decreased respectively to 95%, 91%, and 79% at the end of processing (Fig. 1g; Fig. S2c, see online supplementary material). Compared to fresh samples, the content of all PLs species decreased in dried samples (Fig. 1g; Fig. S2d–I, see online supplementary material). The content of the main PS forms, 42:2, 42:3, decreased by 97% in the dried samples (Fig. 1g; Fig. S2d, see online supplementary material). Meanwhile, the content of the main PG forms, 34:2, 34:1, decreased by 74%, 72% at the end of processing (Fig. 1g; Fig. S2e, see online supplementary material). Furthermore, the main molecular forms of PC, PE, PI, and PA were 34:3 and 34:2, and the contents of the main PC forms, 34:3, 34:2, decreased by 89% and 90%, respectively, in the dried samples (Fig. 1g; Fig. S2f–i, see online supplementary material). The contents of the main PE forms, 34:3 and 34:2, showed, respectively, a 90% and 86% decrease in the dried samples (Fig. 1g; Fig. S2g, see online supplementary material). The contents of the main PI forms, 34:3 and 34:2, decreased by 81% and 80%, respectively, in the dried samples (Fig. 1g; Fig. S2h, see online supplementary material). The contents of the main PA forms, 34:3 and 34:2, decreased by 86% and 85%, respectively, in the dried samples (Fig. 1g; Fig. S2i, see online supplementary material).

The article "Lipidomics, transcription analysis, and hormone profiling unveil the role of CsLOX6 in MeJA biosynthesis during black tea processing" was retracted in 2024. Reasons: no approval from a third party; concerns about the data; concerns about the authorship.

### Lysophospholipid profiles in the leaves during black tea processing

Three types of lysophospholipids, lysophosphatidylcholine (LPC), lysophosphatidylethanolamine (LPE), and lysophosphatidylglycerol (LPG), were detected in tea leaves (Fig. 1e; Figs S4 and S5, see online supplementary material). LPG showed the highest content among them and it accounted for 7% of the glycerolipids in fresh leaves. Meanwhile, the percentage of LPG increased during black tea processing up to 14% in dried leaves (Fig. S5, see online supplementary material). However, the content of LPG decreased during black tea processing and down to the original 0.2% in dry leaves (Fig. 1e). The proportions of LPC and LPE were very low and amounted to less than 0.1% in fresh leaves (Fig. S5, see online supplementary material). While their proportions increased, their contents decreased during processing with the total of LPC and LPE contents, respectively, dropping to 40% and 25% in the dried samples compared to that of fresh samples (Fig. 1e; Fig. S5**,** see online supplementary material). The content of the main LPG species, 16:1, also decreased by 82% during processing, a similar trend being observed for the other LPG species, 16:0, 18:1, 18:2, and 18:3 as well (Fig. 1g; Fig. S4, see online supplementary material). Different than for LPG, 16:0 was the LPC and LPE main species, with most LPC and LPE species showing similar trends with the total LPC or LPE, except for 18:3 LPC content, which decreased during processing (Fig. 1g; Fig. S4, see online supplementary material). Meanwhile, the 16:0 forms of LPC and LPE increased, respectively, almost 4- and 1.5-fold during the fermentation step (Fig. 1g; Fig. S4, see online supplementary material).

The differences in glycerolipid contents among the samples were analysed via principal component analysis (PCA) (Fig. 1f). The PCA model explained more than 62% (R2) of the differences and predicted more than 46% (Q2) of the total variance. Principal component 1 (PC1) described the separation of lipids in different stages during black tea processing, whereas principal component 2 (PC2) explained the effects of processing. Lipids from the fermentation and dried leaves were apparently separated into two groups, while the profiles from fresh and rolling leaves were clustered into a single group (Fig. 1f).

### Neutral lipid profiles in the leaves during black tea processing

Neutral lipids were determined by gas chromatography flame ionization detection (GC-FID) and thin layer chromatography (TLC). The main fatty acids detected in tea leaves were C16:0, C18:0, C18:1, C18:2, and C18:3 and they accounted, respectively, for 28%, 4%, 10%, 27%, and 31% in fresh leaves (Fig. 2; Fig. S6, see online supplementary material). Meanwhile, there was no significant change in the proportions of total fatty acids during processing (Fig. S6a, see online supplementary material). However, a sharp drop was noticed in the content of total fatty acids C16:0, C18:0, C18:1, C18:2, and C18:3, respectively, by 68%, 74%, 80%, 72%, and 76% in dried samples compared to fresh ones (Fig. 2a). Moreover, the content of total fatty acid decreased 73% in dried samples (Fig. 2a). To further explore other neutral lipids profiles, we performed TLC (Fig. 2b). Because only traces of diacylglycerol (DAG) were detected, only triacylglycerols (TAG) and free fatty acids (FFA) were quantitated by GC-FID (Fig. 2c and d). The results showed that the total contents of TAG and FFA fatty acids decreased during processing, respectively, by 91% and 38% in dried samples compared to fresh ones (Fig. 2c and d). Meanwhile, C16:0 from TAG and FFA was the highest form and accounted, respectively, for 44% and 61% in fresh leaves. The content of all TAG and FFA fatty acids declined during processing, except for FFA C16:0 and C18:0 forms (Fig. 2c and d; Fig. S6b and c, see online supplementary material). The proportion of all fatty acids in TAG and FFA remained virtually stable during processing (Fig. S6b and c, see online supplementary material).

The article "Lipidomics, transcription analysis, and hormone profiling unveil the role of CsLOX6 in MeJA biosynthesis during black tea processing" was retracted in 2024. Reasons: no approval from a third party; concerns about the data; concerns about the authorship.

**Figure 2:** Fatty acid profiling during black tea processing. **(a)** Compositions and contents of fatty acids from leaves during black tea processing. **(b)** TLC separation of TAGs from leaves during black tea processing. **(c)** Changes of TAG contents and compositions in leaves during black tea processing. **(d)** Changes of FFA contents and compositions in leaves during black tea processing. Means + SE values are shown (*n* = 3). Significance levels are as follows: ^*^P < 0.05 and ^**^P < 0.01 (Student’s *t*-test).

### Hormone profiles in the leaves during black tea processing

Hormone determination showed that JA and MeJA are produced in high amounts during black tea processing, and especially with respective increases of almost 6- and 3-fold during fermentation (Fig. 3). Meanwhile, the JA derivative jasmonoyl-isoleucine (JA-Ile) decreased during processing, except during rolling, and then dropped 42% during drying compared to freshly harvested leaves (Fig. 3). In addition to citric acid (CA), methyl citric acid (MeCA), we also analysed the contents of other hormones: salicylic acid (SA), methyl salicylate (MeSA), abscisic acid (ABA), indole-3-acetic acid (IAA), methyl indole-3-acetic acid (MeIAA), benzylaminopurine (BA), indole-3-butyric acid (IBA), and zeatin. The contents of SA, IAA, BA, and MeCA increased during the withering step and then decreased in the subsequent step by, respectively, 31%, 70%, 85%, and 85% during drying (Fig. 3). However, the contents of MeSA and IBA-2 declined during processing, culminating with a final decrease of 86% and 93% in dried leaves, respectively (Fig. 3). Meanwhile, ABA and CA levels were steady during most of the processing but decreased, respectively, 54% and 75% during drying (Fig. 3). Both MeIAA and zeatin were largely synthesized during processing with their respective contents upping almost 12- and 1.6-fold during fermentation (Fig. 3). On the other hand, the MeIAA level increased 6.5-fold, and zeatin decreased 16% during drying compared to fresh samples (Fig. 3).

The article "Lipidomics, transcription analysis, and hormone profiling unveil the role of CsLOX6 in MeJA biosynthesis during black tea processing" was retracted in 2024. Reasons: no approval from a third party; concerns about the data; concerns about the authorship.

**Figure 3:** Hormones levels in leaf samples during black tea processing. Means ± SD values are shown (*n* = 3). Significance levels are as follows: ^*^P < 0.05, and ^**^P < 0.01 (Student’s *t*-test). ABA, abscisic acid; BA, benzylaminopurine; CA, citric acid; IAA, indole-3-acetic acid; IBA, indole-3-butyric acid; JA, jasmonic acid; JA-Ile, jasmonoyl-isoleucine; MeCA, methyl citric acid; MeIAA, methyl indole-3-acetic acid; MeJA, methyl jasmonate; MeSA, methyl salicylate; SA, salicylic acid.

### Expression profiles of genes involved in the MeJA synthesis pathway in leaves during black tea processing

Although MeJA is synthesized from lipid degradation, the profiles of genes involved in this pathway during black tea processing remain unknown. We analysed the transcription profiles of *phospholipase A* (*PLA*), *LOX*, *AOS*, *AOC*, *OPR*, *ACX*, *JMT*, *hydroperoxide lyase (HPL),* and *alcohol dehydrogenase (ADH)* in the MeJA synthesis pathway via RNA-Seq and qRT-PCR during different stages of black tea processing (Fig. 4). Results confirmed that most genes were expressed during black tea processing, and that RNA-Seq analysis was comparable with qRT-PCR data (Fig. 4b and4c; Fig. S7 and Table S1, see online supplementary material). However, not all genes were highly expressed during processing: 79, 14, 1, 4, 10, 9, 10, 3, and 23 genes were annotated as *PLA, LOX, AOS, AOC, OPR, ACX, JMT, HPL,* and *ADH*, respectively (Fig. 4b; Table S1, see online supplementary material). Among them, *TEA010910* of *PLA*, *TEA012289* of *LOX*, *TEA001041* of *AOS*, *TEA012644* of *AOC*, *TEA026806* of *OPR*, *TEA019216* of *ACX*, *TEA015791* of *JMT*, *TEA008699* of *HPL*, and *TEA024897* of *ADH* displayed the highest expression levels in fresh leaves than the other isoforms (Fig. 4b). All of these genes were clearly downregulated during processing, except for *AOS* (*TEA001041*) and *OPR* (*TEA026806*), which first declined and then increased during fermentation. On the other hand, the expression levels of *JMT* (*TEA015791*) and *HPL* (*TEA008699*) first increased during withering and rolling and then declined during fermentation (Fig. 4b and4c; Fig. S7, see online supplementary material). Meanwhile, *PLA* (*TEA010910*) transcriptional activity decreased approximately 79%, and *LOX* (*TEA012289*), *AOC* (*TEA012644*), *ACX* (*TEA019216*), and *ADH* (*TEA024897*) expression decreased, respectively, 76%, 85%, 50%, and 80% during fermentation (Fig. 4b). Obvious differential expression was observed during processing for *AOS* (*TEA001041*), which was almost 11-fold in upregulated during fermentation, and for *JMT* (*TEA015791*) and *HPL* (*TEA008699*), which were, respectively, induced almost 1.8- and 2-fold during rolling.

The article "Lipidomics, transcription analysis, and hormone profiling unveil the role of CsLOX6 in MeJA biosynthesis during black tea processing" was retracted in 2024. Reasons: no approval from a third party; concerns about the data; concerns about the authorship.

**Figure 4:** Expression profiles of genes involved in the MeJA synthesis pathway during black tea processing. **(a)** The main pathway of jasmonate biosynthesis. 13-HPOT, 13(S)-hydroxy linolenic acid; ACX, acyl-CoA-oxidase; ADH, alcohol dehydrogenase; AOC, allene oxide cyclase; AOS, allene oxide synthase; HPL, hydroperoxide lyase; JA, jasmonic acid; JMT, carboxyl methyltransferase; LOX, lipoxygenase; MeJA, methyl jasmonate; OPC, 3-oxo-2-(2-pentenyl)-cyclopentane-1-octanoic acid; OPDA, 12-oxo-phytodienoic acid; OPR, OPDA reductase; PLA, phospholipase A . **(b)** Gene transcription of MeJA synthesis pathway during black tea processing. Expression values are presented as log2 (FPKM). **(c)** qRT-PCR confirmation of transcriptome. Data are shown as means ± SD from three independent experiments. Significance levels are as follows: ^*^P < 0.05 and ^**^P < 0.01 by the Student’s *t*-test.

In contrast to *TEA010910*, some other *PLA* isoforms (*TEA030352*, *TEA003141*, *TEA030444*, and *TEA031550*) were induced in fermented samples (5-, 7-, 3.5-, and 10-fold, respectively) compared with fresh leaves (Fig. 4b and4c). The expression levels of other *PLA* isoforms (*TEA007581, TEA030027, TEA019960, TEA009379, TEA006034,* and *TEA021525*) increased at the withering, rolling, and fermentation stage to fresh samples, and were induced, respectively, about 6-, 4-, 3-, 2-, 2.5-, and 3-fold in the rolling stage compared to fresh samples (Fig. 4b). The transcription levels of the remaining *PLAs* genes were either consistently low or virtually steady during black tea processing. The expression of *LOX* (*TEA009423*) increased during black tea processing with a 1.7-fold induction in fermented leaves compared to fresh ones. Meanwhile, the expression of most of the remaining *LOX* genes first increased and then declined during fermentation, except for *LOX* (*TEA025499*), which showed the opposite trend and was repressed about 54% in the rolling stage compared to fresh leaves (Fig. 4b and c; Fig. S7, see online supplementary material). *AOC* (*TEA020075*) had a similar expression trend during black tea processing compared to the main *AOC* (*TEA012644*) and decreased 72% during fermentation. In the meantime, *AOC* (*TEA011480*) was downregulated 32% during rolling, with a clear ‘V’ expression trend during processing, an opposite trend comparted to another *AOC* isoform (*TEA001905*), which was upregulated almost 2-fold in the rolling step (Fig. 4b). Most of the *OPR* genes (*TEA025907, TEA026804, TEA033668, TEA027519*, and *TEA022667*) were repressed during black tea processing, except for *OPR* (*TEA029800*, *TEA020350*), whose expression levels for both first increased 49% at withering and then declined at fermentation (Fig. 4b). JA was produced by three steps of oxidation by ACX. Contrasting the main downregulated *ACX* (*TEA019216*), another *ACX* gene (*TEA007262*, *TEA017099*) was upregulated during black tea processing and increased, respectively, almost 22- and 2.5-fold in the fermentation leaves compared to fresh leaves. The expression of two other *ACX* genes (*TEA009681* and *TEA014338*) fluctuated during processing (Fig. 4b). *JMT* is a key gene for MeJA biosynthesis. Several *JMT* genes (*TEA028050, TEA028051, TEA015176*, and *TEA031418*) showed the similar expression patterns to the main *JMT* gene (*TEA015791*) during black tea processing, except for *TEA032708*, which was downregulated by 93% during fermentation (Fig. 4b). On the other hand, the activity levels of some *JMT* homologues (*TEA032424*, *TEA031962*, and *TEA030024*) were very low throughout (Table S1, see online supplementary material). The *HPL* and *ADH* genes belong to a branch of MGDG or DGDG degradation, which can produce C6- and C9-volatiles, such as 3-hexenal and n-nonanal. The expression level of some *HPL* genes (*TEA030439*, *TEA014723*) in all processing steps of black tea processing was lower than that of fresh samples, and fluctuated during processing, and terminated with decreased levels, respectively, at 7% and 77% in dried leaves (Fig. 4b). The expression of most ADH genes was lower during withering and rolling compared to fresh samples, except for *TEA032966*, *TEA015686*, and *TEA006862*, which increased approximately 21%, 33%, and 48% during rolling and then decreased during fermentation (Fig. 4b). All in all, we characterized the expression patterns of genes during black tea processing and identified several ones that were significantly induced post-harvest and may play relevant roles to develop the rich aromas that contribute to high-quality beverages.

The article "Lipidomics, transcription analysis, and hormone profiling unveil the role of CsLOX6 in MeJA biosynthesis during black tea processing" was retracted in 2024. Reasons: no approval from a third party; concerns about the data; concerns about the authorship.

### Suppression of CsLOX6 expression leads to a reduction of MeJA contents

Because a large amount of MeJA is produced in the fermentation stage and only *CsLOX6* (*TEA009423*) still has a continuous high expression in the fermentation stage, we transfected buds with *CsLOX6* (*TEA009423*) *asODN* (Fig. 5a). This LOX homologue was chosen for functional characterization because it is the only one that consistently showed high expression levels in the buds as well as young and mature leaves, which are often harvested for black tea processing, and was induced during all processing stages (Fig. 4b and5b; Fig. S7, see online supplementary material). Compared to the transfection agent (80 mM sucrose solution) and the sense oligonucleotide transfection (sODN in 80 mM sucrose) controls, the *CsLOX6 asODN* treatment efficiently and significantly reduced about 32% of *CsLOX6* transcript levels (Fig. 5c). Further metabolite analysis showed that *asCsLOX6* significantly reduced the content of JA and its natural analogues, OPDA, dnOPDA, MeJA, and JA-Ile, which respectively decreased 27%, 24%, 33%, 38%, and 34% by *asCsLOX6* transfection compared to the controls (Fig. 5d). Moreover, MeSA and SA contents detected in the same *asCsLOX6* line increased 47% and 10%, respectively, and ABA decreased about 55% in the *asCsLOX6* line compared with control (Fig. 5d). The reduction of JA analogue was confirmed by qRT-PCR of the transcriptional repression of genes involved in the MeJA synthesis pathway (Fig. 5e). *asODN*-transfected buds showed significant reduced 57%, 50%, 29%, and 57% transcript contents, respectivel,y of *CsAOS*, *CsAOC1*, *CsACX1*, and *CsJMT1* compared to the controls, but it did not affect the expression of *CsPLA1* (Fig. 5e). Meanwhile, *CsHPL1* expression also decreased by 69% in the *asODN* line, which was supported by the volatile contents in *asCsLOX6* compared to the control. Indeed, GC–MS/HS-SPME analysis showed that the contents of most volatiles, such as hexanal and 2-hexenal, in *asCsLOX6* line were lower than that of the control line (Fig. S8, see online supplementary material).

**Figure 5:** *CsLOX6* potentially affects MeJA biosynthesis. **(a)** Antisense knockdown of *CsLOX6* by treatment with oligodeoxynucleotides (asODN). **(b)** Tissue expression of *CsLOX6*. B, apical bud; Fl, flower; Fr, fruit; L1, young leaf; L2, mature leaf; L3, old leaf; R, root; S, stem. **(c)** Effects of asODN treatment on *CsLOX6* mRNA levels. Relative transcript levels were determined by quantitative real-time PCR. **(d)** Effects of asODN treatment on hormone levels. Abbreviations: OPDA, 12-oxo-phytodienoic acid; dnOPDA, dinor-12-oxo-phytodienoic acid. **(e)** Effects of asODN treatment on transcription of genes related to the MeJA synthesis pathway. Data are shown as means ± SD from three independent experiments. Significance levels are as follows: ^*^P < 0.05 and ^**^P < 0.01 by the Student’s *t*-test.

## Discussion

The composition and content of lipids in cellular membranes, plant tissues, and organisms vary significantly [13, 21, 22]. In tea, lipids play a crucial role in conferring unique characteristics to the beverage as they serve as precursors of aroma compounds [13]. Many lipids, including PC, PE, PI, and PA species, participate extensively in stress responses in plants [9, 23–25]. During black tea processing, the structural lipids in the leaves undergo widespread damage due to various factors such as wounding, dehydration, heat, and enzymic reactions [4, 10]. As a result of the processing, there is a decrease in the levels of structural lipids GLs and PLs, accompanied with different main lipids species reduced, such as 34:3, 36:6 forms DGDG. These observations suggest that lipids undergo oxidation and degradation in tea leaves during processing, which is also seen during wound response [26]. However, unlike wounded leaves in plants, TAG profiling kept a declining trend in black tea processing and wounded and detached tea leaves could not transport TAG to the area around the wounded region to conserve fuel TAG. This is achieved through the conversion of PA and PC into TAG via diacylglycerol intermediates, serving as a transient buffer for acyl chains that are present in excess [27]. These observations highlight the intricate changes in lipid composition and metabolism during black tea processing.

The article "Lipidomics, transcription analysis, and hormone profiling unveil the role of CsLOX6 in MeJA biosynthesis during black tea processing" was retracted in 2024. Reasons: no approval from a third party; concerns about the data; concerns about the authorship.

Our data, along with published studies, support the notion that there is a significant production of JA and MeJA during black tea processing [3]. Morevoer, JA and MeJA show an inverse trend with SA and MeSA, particularly during the rolling step, which is similar to the early wound response in rice [28]. There is no significant change in ABA levels in plucked tea leaves compared to fresh or fermented tea leaf samples, showing a difference with ABA accumulation in *Arabidopsis* upon wounding [29]. In black tea processing, excessive injured and detached tea leaves experience a reduction in IAA levels and an increase in MeIAA levels. Additionally, the precursor of auxin, IBA, undergoes a reduction during processing, as it is converted to IAA through peroxisomal β-oxidation. This phenomenon is different from activating cytokinin and auxin biosynthesis in potato tubers upon slight wounding [30]. During tea processing, the levels of the cytokinin analogue, benzylaminopurine (BA), are found to be induced during the withering step but suppressed during the rolling, fermentation, and drying steps. In contrast, the levels of the cytokinin zeatin increase during processing, except for a significant reduction observed in dried leaves. Interestingly, the levels of endogenous citric acid (CA) remain relatively constant during black tea processing, except for a significant reduction observed in dried leaves. However, the methylated forms of CA, MeCA, show a reduction in levels during processing, except for a slight elevation during withering. All hormones, including JA, SA, their methylations, as well as ABA and IAA, can potentially be produced in detached tea leaves. The levels of JA, SA, and their methylations in detached tea leaves are consistent with those found in wounded leaves. On the other hand, ABA and IAA were mainly produced in wounded plant leaves and showed distinct changes during tea processing. Moreover, excessive mechanical damage to leaves, for rolling, can result in the change of pathway involved in IAA synthesis. Those observations provide insights into the hormonal dynamics during tea processing, suggesting possible roles of specific hormones in different stages of tea production.

The article "Lipidomics, transcription analysis, and hormone profiling unveil the role of CsLOX6 in MeJA biosynthesis during black tea processing" was retracted in 2024. Reasons: no approval from a third party; concerns about the data; concerns about the authorship.

The expression of genes *PLA, LOX, AOS, AOC, OPR, ACX, JMT, HPL,* and *ADH* involved in MeJA biosynthesis has been shown to be associated with both biotic or abiotic stresses responses in plants [16, 17, 31–35]. When considering their expression in detached leaves during black tea processing, main homologous genes in lipid degradation pathway present a downregulated trend and non-primary genes tend to be a little high or fluctuation expression in black tea processing. The expression difference in black tea processing between primary and non-primary genes perhaps complements each other to repair the broken function and restores the fragmented signal transduction in detached and excessively damaged tea leaves. In the meantime, factors such as functional enzyme from internal cells interacting with the stressed external environment further weaken the leaves function during black tea processing. Moreover, a clear opposite trend is observed between the expression of the main *CsHPL (TEA008699)* and *CsAOS (TEA001041)* genes throughout tea processing compared to fresh leaves, which influences the direction of lipid derivative flow and decides MeJA production during black tea processing. Additionally, the expression of the main Cs*JMT (TEA015791)* gene correlates with the content of its product, MeJA, during black tea processing. The coordinated expression of the main *CsHPL (TEA008699), CsAOS (TEA001041)*, and Cs*JMT (TEA015791)* result in high production of MeJA during black tea processing. These findings highlight the complex regulation of MeJA biosynthesis and its involvement in black tea processing responses.

The comprehensive analysis combining lipidomics, hormone metabolism, and transcriptome data has provided valuable insights into the key genes and pathways involved in aroma-related volatiles during black tea processing. The findings support the notion that there is a decrease of structural lipids GLs, PLs, and stored TAG, accompanied with different main lipids species reduced, such as 34:3, 36:6 forms of DGDG, during black tea processing. The degraded lipids are transformed into the production of substantial amounts of MeJA and JA, accompanied with the decreased SA, MeSA, IAA, and BA and increased zeatin. Moreover, the main homologous genes in lipid degradation pathway present a downregulated trend except for *AOS (TEA001041)* and *OPR (TEA026806)* and non-primary genes tend to a little high or fluctuation expression in black tea processing further supports these observations. The coordinated expression of the main *CsHPL (TEA008699), CsAOS (TEA001041)*, and Cs*JMT (TEA015791)* result in the high production of MeJA during black tea processing. This suggests that the interplay between these genes potentially determines the direction of lipid derivative flow in MeJA metabolism during tea processing. One important finding is that knock-down of *CsLOX6* significantly reduced the level of jasmonates and expression of downstream genes, accompanied with SA, MeS level rising, and ABA declining. This work lays a solid theoretical foundation for galactolipids, mainly 34:3/36:6/36:3 DGDG and 36:6/36:5/36:4 MGDG, are transformed into MeJA in black tea processing, accompanied with hormonal dynamics regulation and coordinated expressed *CsHPL (TEA008699), CsAOS (TEA001041)*, and *CsJMT (TEA015791)* control. These results have significant implications for future studies in black tea processing.

The article "Lipidomics, transcription analysis, and hormone profiling unveil the role of CsLOX6 in MeJA biosynthesis during black tea processing" was retracted in 2024. Reasons: no approval from a third party; concerns about the data; concerns about the authorship.

## Materials and methods

### Plant material and sampling

The black tea processing method followed a similar procedure described in previous reports [11, 36]. Tea resources (*C. sinensis* cv. Shuchazao), aged eight years, were acquired from the Guohe tea plantation in Hefei, Anhui, China (latitude 31.3^o^N, longitude 117.2°E). Fresh tea leaves were harvested on 1 August when temperatures ranged between 26–32°C with a relative humidity at 53%. A portion of the freshly harvested material was immediately immersed in liquid nitrogen, while another part underwent an immediate withering process that involved spreading the plucked leaves evenly and allowing them to wither for 12 hours. Subsequently, the withered leaves were manually rolled for 30 min. To initiate fermentation, the rolled leaves were subjected to a heat-moisture treatment at 90% humidity for 3 hours. Following fermentation, the material was dried for ten minutes in a 90°C oven. Throughout each step, samples were collected and rapidly frozen in liquid nitrogen, then stored at −80°C for future analysis.

### Chemicals

Chloroform, acetic acid, methanol, hexane, butylated hydroxytoluene, sulfuric acid, isopropanol, acetone, diethyl ether, iodine, toluene, hydrochloric acid, acetone, formic acid, heptane, and acetonitrile were sourced from Sinopharm Chemical Reagent (Hefei, China). C17:0 fatty acid (Sigma-Aldrich) was employed as an internal standard. All reagents and solvents utilized in this study were of analytical or HPLC grade and were procured from commercial suppliers. Aqueous solutions were prepared using freshly double distilled water (ddH_2_O) exclusively.

The article "Lipidomics, transcription analysis, and hormone profiling unveil the role of CsLOX6 in MeJA biosynthesis during black tea processing" was retracted in 2024. Reasons: no approval from a third party; concerns about the data; concerns about the authorship.

### Lipid analyses

Galactolipids, phospholipids, triacylglyceride (TAG), free fatty acid (FFA), and total fatty acid analysis was similar to the protocol as published [37, 38]. Tea leaves powder was pretreated using isopropyl alcohol at 75°C, supplemented with 0.01% butylated hydroxytoluene (BHT) for 5 min, and mixed with extract solvent of chloroform, methanol, and water (10/10/1) with 0.025% of BHT. Subsequently, the leaves were shaken for 30 min and the supernatant was evaporated. The final residual was dissolved in 1 mL chloroform for galactolipids, phospholipids analysis. Thin layer chromatography (TLC) analysis of the composition of galactolipid and phospholipid, the extracted solvent mixture of methanol, chloroform, and formic acid (20:10:1, v/v/v), separated solvent of acetone, toluene, and water (91:30:7.5, v/v/v), and visual reagent iodine were used as previously described [37]. TAG and FFA analysis used 30-mg samples to mix 4 M HCl for 30 min and then boiled for another 10 min. Subsequently, the mixture was vortexed with 4 mL of hexane and isopropanol mixture (3:2, v/v) and the supernatant was collected for N_2_ evaporation. The final residual was dissolved in 50 μL of hexane for analysis. Total fatty acid profiles analysis used the sulfuric acid/methanol method. A mixture of ground samples (50 mg) and 1 mL 2.5% sulfuric acid in methanol was heated at 90°C for 30 minutes then mixed with 0.5 mL of water and 0.7 mL of heptane and the top layer collected for analysis.

### Hormone quantification

The previously established procedure was used for hormones analysis [39]. Samplespowder was extracted and then vortexed with a cold mixture of acetonitrile, water, and formic acid (25: 75: 0.1, v/v/v). After sonicating in a cold water bath for 20 min and rotating extraction at 4°C for 16 h, the supernatant was collected and the pellets were extracted again. The combined supernatants were dried under N_2_ evaporation and the remaining residue was dissolved in methyl alcohol for LC–MS/MS analysis. An Agilent 1290 HPLC system coupled with a reversed-phase column (Poroshell 120 SB-C18, 2.1 × 150, 2.7 μm) was equipped with an AB Qtrap6500 mass spectrometer with electrospray ionization (ESI) as the ion source. Mobile phase A and B contained 0.1% formic acid in distilled water and methanol, respectively. The flow rate of the mobile phase was 0.25 mL/min and gradient elution procedures were set as follows: 40% B (12 min), 100% B (2 min), and 40% B (8 min). All assays were performed with three biological replicates.

The article "Lipidomics, transcription analysis, and hormone profiling unveil the role of CsLOX6 in MeJA biosynthesis during black tea processing" was retracted in 2024. Reasons: no approval from a third party; concerns about the data; concerns about the authorship.

### RNA isolation and cDNA library construction for Illumina sequencing

Following the provided instructions, an RNA kit (Biotech, Beijing) was used to extract the RNA from different stages of black tea processing. Based on the methods established in our lab, 0.5–2 μg RNA was used for reverse transcription and library construction. Seven GB of RNA-Seq data were acquired for each sample by sequencing on an Illumina HiSeq2500 platform of BGI Shenzhen Biotechnology. eXpress (Trinity, Broad Institute) was employed to calculate fragments per kilobase of exon model per million mapped fragments (FPKM) and transcripts per million (TPM). The subsequent differential gene expression (DGE) analysis method was similar to a previous publication [11]. For MeJA biosynthesis analysis in black tea processing, relevant data were extracted from the RNA-Seq Atlas data. Heatmaps were generated with TBtools for visualization and analysis purposes (https://github.com/CJ-Chen/TBtools).

### Quantitative RT-PCR (qRT-PCR) analysis of gene expression

qRT-PCR analysis was conducted following a previously described method [11]. The RNA exraction method followed the TRIzol reagent manufacturer’s instructions. Separated RNA was digested with RNase-free DNaseI (Promega, Madison, WI, USA) to remove the DNA contamination. The purified RNA in each tea leaf was determined by a NanoDrop ND-2000 UV spectrophotometer (Thermo Scientific, USA) and then carried out for first-strand cDNA synthesis using the SuperScript IV (Invitrogen) kit based on the written instruction. Each cDNA sample was diluted 50-fold and added 2 μL of 100 ng into the PCR reaction (20 μL), to which was supplied 10 μL Power SYBR Master Mix (Applied Biosystems), 2 μL primer mix (10 umol/uL), and 2 μL primer mix (10 umol/uL). iQ5 Real Time PCR System from Bio-Rad was used to perform the PCR reaction. The housekeeping gene *CsACTIN (TEA019484.1)* was used to normalize the relative expressed level. All primers are listed in Table S1 (see online supplementary material).

### Antisense knockdown of CsLOX6 in tea shoot tips

The infiltrated suppression experiment followed similar previously established methods [11, 36]. Soligo software (http://sfold.wadsworth.org/cgi-bin/soligo.pl) was used to screen the interested target and design the oligodeoxynucleotide (ODN) sequences. The tea of *C. sinensis* cv. Shuchazao was inserted in 80 mM sucrose solution containing 700 μM of ODN to perform the ODN-based antisense (*asODN*). The *CsLOX6* (*TEA009423*) *asODN* buds were harvested for gene expression check after 3 days treatment.

The article "Lipidomics, transcription analysis, and hormone profiling unveil the role of CsLOX6 in MeJA biosynthesis during black tea processing" was retracted in 2024. Reasons: no approval from a third party; concerns about the data; concerns about the authorship.

### Extraction of volatiles using HS-SPME (headspace solid-phase microextraction)

The sealed vial (25 ml) containing 0.5 g of samples was equilibrated in water at a temperature of 65°C for 5 min. A hand-held SPME fiber with a DVB/CAR/PDMS coating (50/30 μm, Supelco, St Louis, MO) was reconditioned in the GC injector port at 250°C for 5 min and then inserted into the vials. The fibers were exposed to the headspace for 1 h of extraction time. Subsequently, the needle was directly inserted into the injection port of Agilent 7890A GC–MS coupled with a 7000D triple quadrupole mass spectrometry (GC/MS/MS) system (Agilent, Santa Clara, CA, USA) and a DB-5MS capillary column (30 m × 0.25 mm × 0.25 μm film thickness). High purity helium was at a flow rate of 1 mL/min. The injector temperature was maintained at 250°C in the splitless mode. The oven temperature was initially held at 50°C for 3 min, and reached the temperature of 250°C by a rate of 5°C/min increased, which was held for 5 min. Each sample performed technical triplicates and ethyl decanoate (0.01%) was served as internal standard. An established standard substance or the NIST database was used to identify the chemicals compounds, following a previously described method [40].

### Statistical analyses

A minimum of three independent experiments was recorded for the data and a Student’s *t*-test was performed to assess the statistical significance of the results. The confidence limit 95% represents statistical significance between two-tailed data. SIMICA (v.15.0) software was employed to conduct the principal component analysis (PCA).

## Acknowledgements

We thank Prof. Ruth Welti and Ms Mary Roth at Kansas State University for assistance on lipid metabolite profiling and data analysis, Mrs Ying Huang at Anhui Agricultural University for her assistance with qRT-PCR analyses and sample collection, and Xiongyuan Si at Anhui Agricultural University for technical support in volatile flavor analysis. The authors also thank Prof. Zhao’s lab members for assistance with experiments and data analyses and Vagner’s grammar modification. This work was supported by High Level Research Fund for Qualified People of Henan University of Technology (2021BS017), the Key Research and Development (R&D) Program of Anhui Province (18030701155), the National Key Research and Development Program of China (2018YFD1000601).

## Author contributions

G.Z. conceived the project and supervised this study. G.Z., J.W., L.L., and D.C. performed the experiments. G.Z., J.W., L.L., collected samples and performed the lipidomics analysis. D.C. analysed the gene transciptional expression. G.Z. wrote and edited the manuscript. All authors read and approved the final manuscript.

The article "Lipidomics, transcription analysis, and hormone profiling unveil the role of CsLOX6 in MeJA biosynthesis during black tea processing" was retracted in 2024. Reasons: no approval from a third party; concerns about the data; concerns about the authorship.

## Data availability

All relevant data in this study are provided in the article and its supplementary data files.

## Conflict of interest statement

All authors declare that they have no competing interests.

## Supplementary data

Supplementary data is available at *Horticulture Research* online.

## Supplementary Material

Web_Material_uhae032
